The article "A Rumor Detection Method from Social Network Based on Deep Learning in Big Data Environment" was retracted in 2023. Reasons: signs of a paper mill; compromised peer review; unreliable results or conclusions.

# A Rumor Detection Method from Social Network Based on Deep Learning in Big Data Environment

**DOI:** 10.1155/2022/1354233

**Published:** 2022-03-28

**Authors:** Junjie Cen, Yongbo Li

**Affiliations:** ^1^College of Computer Science and Technology, Henan Institute of Technology, Xinxiang, Henan 453002, China; ^2^College of Computer and Information Engineering, Henan Normal University, Xinxiang, Henan 453002, China

## Abstract

Aiming at the lack of feature extraction ability of rumor detection methods based on the deep learning model, this study proposes a rumor detection method based on deep learning in social network big data environment. Firstly, the scheme of combining API interface and third-party crawler program is adopted to obtain Weibo rumor information from the Weibo “false Weibo information” public page, so as to obtain the Weibo dataset containing rumor information and nonrumor information. Secondly, the distributed word vector is used to encode text words, and the hierarchical Softmax and negative sampling are used to improve the training efficiency. Finally, a classification and detection model based on the combination of semantic features and statistical features is constructed, the memory function of Multi-BiLSTM is used to explore the dependency between data, and the statistical features are combined with semantic features to expand the feature space in rumor detection and describe the distribution of data in the feature space to a greater extent. Experiments show that when the word vector dimension is 300, compared with the compared literature, the accuracy of the proposed method is improved by 4.232% and 1.478%, respectively, and the F1 value of the proposed method is improved by 5.011% and 1.795%, respectively. The proposed method can better extract data features and has better rumor detection ability.

## 1. Introduction

With the development of time and the progress of science and technology, Internet technology has gradually entered thousands of households. As one of Web2.0 (such as Weibo, twitter, wechat, and other platforms), social networks have also developed at an amazing speed [1–3]. Among them, Weibo has quickly won people's favor with its fast and convenient content form and information interaction, which can be widely spread in the society, and has a profound impact on people's living conditions, daily travel, and even all aspects [4–7].

The amount of information on the Internet is very complex, and every user can access an astonishing number of articles or posts through the Internet. At the same time, due to the low threshold for the use of social networks and the lack of an effective way of audit and supervision, it provides convenience for criminals. Criminals can use the characteristics of human nature to spread false information and create fear to achieve their own purposes [8–10]. In addition, ordinary people may also publish their hearsay and shadowy information to social media for verification, which will lead to the generation and spread of rumors [11–14]. The widely spread rumors are usually very confusing. For the general public, due to the lack of relevant knowledge, they often can only judge the information obtained by relying on their own feelings or past experience and cannot effectively judge the information, which may inadvertently aggravate the spread of rumors. Moreover, there are a large number of unidentified and even contradictory information on the network, which also makes users more prone to anxiety and confusion. With the help of online social media, rumors will spread rapidly [15–18]. These spreading rumors will greatly mislead the people become a potential unstable factor in society and affect the stable operation of economy and society.

The automatic detection of network rumors refers to the comprehensive use of Internet, statistics, machine learning, communication, psychology, and other knowledge to let the machine detect rumors. Compared with the time-consuming and laborious characteristics of manual methods, the automatic detection of rumors can detect network hot events in large quantities in real time, so as to effectively deal with the massive information appearing on the Internet every day [19–21]. In recent years, with the development of big data and artificial intelligence technology, rumor detection ability has also been greatly improved. Most research studies on rumors' detection in social networks are based on deep learning methods [22]. At present, the accuracy of automatic rumor detection cannot reach the manual standard, but this is an important breakthrough in purifying cyberspace.

In order to detect rumors in social networks as soon as possible, Chen et al. [23] proposed an unsupervised learning model combining recurrent neural network and variational autoencoder to learn the network behavior of social network users. By using the significant difference between normal data and abnormal data in the dimensionality reduction process, the error between the output and the target value is compared with the specified threshold to judge whether it is a rumor. Guo et al. [24] proposed a rumor detection model based on hierarchical neural network (HSA-BLSTM) combined with social information. Firstly, a hierarchical two-way long short-term memory model representing learning is established, and then, the weight of the vector is adjusted through the attention mechanism. Wang et al. [25] use multihead self-attention mechanism to detect rumors, extract features from context information, and obtain text local features by CNN. The application of attention mechanism to rumor detection improves the ability of rumor detection. According to the account information of rumor mongering users published in the Weibo rumor refutation, Sun et al. [26] use Weibo API to collect the information of rumor mongering users and use the Weibo information of rumor mongering users, user friend information, and Weibo information published by user friends for Weibo rumor detection. Yongheng Chen et al. [27] proposed a rumor early detection multitask learning (RL_MT_RED) based on reinforcement learning, which describes the closely related rumor detection and position classification problems as a multitask learning and joint learning. RL_MT_RED integrates reinforcement learning to control multitask learning and realizes the dynamic setting of trusted checkpoints. Li et al. [28] proposed a rumor tracking integration model based on deep reinforcement learning (RL-ERT), which aggregates multiple components through the weight adjustment strategy network and uses specific social characteristics to improve the performance of the model. Lin et al. [29] proposed a deep sequence context model for Weibo rumor detection, which considers two important factors of rumor: falsity and influence. Firstly, in order to learn falseness, the hypothesis of word independence is cancelled, and the long-term and short-term memory units are used to capture the two-way sequence context information in the content. Secondly, in order to understand the impact, the deep-seated contextual information is combined with social characteristics to understand the relationship between content and social characteristics. Although these methods have achieved certain results, most of the data feature extraction is not sufficient, which belongs to the shallow extraction of rumor recognition elements, so it cannot further improve the accuracy.

Based on the above analysis, the current research mainly manually establishes semantic features from the text content of rumors, which has the problem of insufficient feature extraction ability. Therefore, a rumor detection method based on deep learning in the social network big data environment is proposed. The main improvements of this study are as follows: using distributed word vector to encode text words, which improves the operation efficiency in the case of a large number of corpus. In the optimization training stage, hierarchical Softmax and negative sampling are used to improve the training efficiency. Specifically, this study constructs a multi-BiLSTM network and statistical feature fusion model to deeply extract text features and improve the classification efficiency. The attention mechanism is introduced to adjust the weight of the vector, which improves the efficiency and accuracy of task processing. Experiments show that the proposed method can better extract data features and has better rumor detection ability.

## 2. Rumor Detection Process Based on Deep Learning

At present, rumor detection is mainly based on traditional machine learning. It usually establishes features manually from the three aspects of rumor text content, communication structure, and credibility. The manually established features are single and the process of establishing features is time-consuming. To solve these problems, this study proposes a Weibo rumor detection model based on deep learning, which automatically extracts the characteristics of rumor by training neural network through rumor Weibo data, so as to realize the detection of Weibo rumor. The overall method flow is shown in Figure 1. The idea of this study is to obtain rumor and nonrumor Weibo data from Weibo platform, establish corpus, filter spam comments, and carry out word segmentation, word vectorization, and other operations. Secondly, the text vector is input into the neural network. In order to get better experimental results, a rumor detection model based on multi-BiLSTM network is proposed in this study. Finally, a comparative experiment is set up to verify the effectiveness of the proposed method in rumor detection.

## 3. Weibo Data Collection and Text Word Vector Training

### 3.1. Construction of Weibo Corpus

To use the massive data of Weibo to study rumors, it is necessary to do a good job in data collection and cleaning. Using the combination of API and third-party crawler program, the Weibo dataset contains rumor information and nonrumor information.

The Weibo open platform provides more than 200 API interfaces, which can download Weibo content, comments, likes, forwards, and other related information. Users can use OAuth2.0 to collect relevant information and build a local database after obtaining authorization. The authorization process of OAuth protocol is shown in Figure 2.

The web crawler program can automatically collect web page information according to the network protocol and crawl from the initial URL. The crawler program uses search engine and web page hyperlink to obtain web page information. This study uses simulated Login technology to obtain deeper information on the page until the crawled data meet the requirements. At present, it is not easy to collect a large amount of Weibo text data, and there are few public text corpora for Weibo. Therefore, when solving the problem of Weibo rumor detection, we usually need to collect our own research corpus. This study selects the scheme of combining API and third-party crawler program to obtain data. The Weibo dataset contains rumor information and nonrumor information.

Sina company directly publishes false Weibo information in the Weibo community management center, so it can directly climb the rumor text on the center page to build a rumor Weibo dataset. This method not only is simple and fast but also avoids the problem of manual annotation and reduces a lot of manpower and time. This study mainly collects 10385 pieces of rumor Weibo information published by the Weibo management center from March 1, 2019, to November 31, 2021. At the same time, it collects the name of the whistleblower Weibo, the link of the whistleblower Weibo, the Weibo name of the whistleblower, and the rumor comments. Then, crawl the normal Weibo, as well as relevant comments and forwarding. Finally, 10385 rumor Weibo and 10759 nonrumor Weibo were collected, respectively, the proportion of training set and test was 9 : 1, and the relevant comments were 158952.

### 3.2. Vector Representation of Text

The word vector generated in the form of one hot is too sparse and has too many invalid positions, which will greatly consume the amount of calculation and the physical memory of the computer in practical application. This study uses distributed word vector to encode words. Word2vcc mainly uses two models: Continuous Bag of Words Model (CBOW) and Skip-Gram model. Figures 3 and 4 show the basic structures of these two models. The input of the model is the effective vector, and then, it will pass through a projection layer. Finally, the data of the output layer are used for softmax regression to obtain the output vector.

The training goal of the CBOW model is to predict the occurrence probability *p*(*w*_*i*_*|w*_*i*−*k*_,…, *w*_*i*−1_, *w*_*i*+_,…, *w*_*i*+*k*_) of the target word according to the context information of the target word. The Skip-Gram model, on the contrary to CBOW, uses the target word to predict the context word in its context, that is, the input is the word vector of a specific word, while the output is the context corresponding to a specific word, and the output size is related to the window size set in advance. CBOW is more suitable for small corpora, while the Skip-Gram model performs better in large data corpora.

### 3.3. Optimization Training

Word2vec implements the optimization algorithm of word vector representation in theory. However, in practical application, the Chinese corpus is very large, and the number of words reaches millions. In the above two models, the whole vocabulary needs to be calculated, which will cause great difficulties in training and calculation. This study uses hierarchical Softmax and negative sampling to speed up the training speed and improve the training efficiency.

#### 3.3.1. Hierarchical Softmax

The essence of hierarchical softmax is to turn the N-classification problem into log(*N*) quadratic classification. In this optimization method, instead of using the traditional DNN network training parameters, Huffiman tree is used to replace the neurons in the hidden and output layer. The leaf node of Hufiman tree plays the role of output neuron. The leaf node is the size of vocabulary, and the internal node of Hufiman tree plays the role of the hidden layer. Taking the CBOW model as an example, the output layer corresponds to a Hufiman tree, which takes the words appearing in the corpus as the leaf node and the word frequency as the weight of the node. For any word in dictionary D, there must be a unique path from the root node to the word in the Hoffman tree. Each branch on the path can be regarded as a binary classification problem. Each classification produces a probability. Multiplying these probabilities can obtain the target probability. Therefore, the output layer is changed from the original model single layer to the Hufiman tree.

#### 3.3.2. Negative Sampling

In the corpus, positive samples are the data samples represented by the current word and its context word, and some context words and current words are randomly generated to form negative samples. Negative sampling is the process of randomly generating context words. When solving the objective function, considering that the central word and its negative sample cannot appear in the training data window at the same time, the probability distribution formula can be understood as the joint probability of the probability that the current word and the negative sample word are not observed in this window. The final optimization objectives are defined as follows:

(1) $$\begin{array}{c} \log\;p\left(w_{t}|c_{t}\right)=\log\;s\left(w_{t},c_{t}\right)+\sum_{k=1}^{K}\log\left(1-s\left(w_{k},c_{t}\right)\right), \end{array}$$

where *w*_*t*_ is the current vocabulary, *c*_*t*_ is the context, and *w*_*k*_ is a random negative sample. Thus, the change from calculating the whole vocabulary to calculating only *K* negative samples is realized, and the time complexity is reduced.

## 4. Classification and Detection Model Based on the Combination of Semantic Features and Statistical Features

The traditional word embedding method realizes the shallow extraction of text features, but the task of rumor detection requires the deep extraction of text features, so as to improve the classification efficiency. With the popularity of deep learning in recent years, the use of deep network to extract rumor features has achieved excellent results, among which the RNN network represented by LSTM is the most common. In this study, multi-BiLSTM network and statistical feature fusion are selected as the network structure of feature extraction. On the one hand, text data have natural serialization characteristics, and LSTM can retain the location information of text. On the other hand, general social media information belongs to typical short text. LSTM uses a gating mechanism to effectively solve the problems of less context information and unclear semantics in short text.

In order to solve the problems of shortage of single microblog content, lack of semantics and inability to integrate global features by simple semantic classification. At the same time, as the current distributed expression of words can bring more semantic information and the training and use of word vectors are becoming more and more standardized, this section proposes based on multifeature fusion. That is, the deep neural network model integrating statistical features and semantic features. The proposed model based on multi-BiLSTM and statistical feature fusion is shown in Figure 5. This study adopts a deep learning model based on the combination of semantic features and statistical features. The first part extracts the semantic features of Weibo. Firstly, the input Weibo data are transformed into time-series data. Multi-BiLSTM has memory function and can find the dependency between data. Therefore, the semantic features that change with time can be learned through the multi-BiLSTM model. This study introduces the attention mechanism to connect different modules and give the weight value to each module in the global scope. The more important the module with high weight value is in feature selection, the lower the value and proportion of the module with low weight value in semantic feature representation. The second part is used to extract the social features based on user information, the social features of communication content and the social features of Weibo content, vectorize the three types of features, splice the vectorized features into a one-dimensional vector, and then map them into a vector with the same dimension as the semantic features through the full connection layer. Finally, the semantic features and statistical features are spliced, and the classification results are obtained through the Softmax layer.

The attention mechanism is introduced into the model because the amount of information contained in the news content is different at different times in the process of news communication. This is related to the communication mode of language. In the early stage of Weibo release, netizens may carry out special communication because of the impossibility or interest of rumors. However, as more and more netizens participate in the discussion of the event, they will doubt the authenticity of the event. At this time, there will be similar “really?” and “impossible?” and other questionable content appears and will also look for official certification. With the development of the event, the news that is finally certified as a rumor will be forwarded with the attitude of popular science. At this time, there will be “this is false” and “deceptive” and other contents. Therefore, in the process of language communication, the importance of message content is different at different time points. For example, in the early stage of forwarding, people only forwarded the interest of the original Weibo, and there is no questioning attitude in the rumor characteristics. Therefore, the message weight of this part can be appropriately reduced. In the middle or late stage of new use communication, the emergence of rumor pattern words brings more semantic information to the forwarding comment content. At this time, the message content can be given a higher weight.

In the model of multi-BiLSTM combined with statistical features, the input of multi-BiLSTM is still represented by paragraph vector divided by time. On the one hand, if each Weibo is input into the model in the form of vector, it is difficult for the model to learn dependent information. On the other hand, the complexity of the model brings difficulties to training and calculation. Therefore, it is necessary to simplify the steps of the model. At the same time, in order to get more semantic information, events are divided into subevents. The length of the model is equal to the number of sub events, and the input of the model is the vector expression of subevents or paragraphs. For a given event *Q*, it is divided into *N* subevents; then, the event representation is *Q*=(*Q*_1_, *Q*_2_, ..., *Q*_*N*_), and the subevent *Q*_*i*_ is a one-dimensional vector with the length of word vector multiplied by the number of words and then multiplied by the number of messages. Each subevent *Q*_*i*_ is used as the input of multi-BiLSTM to obtain the output vector *y*_*i*_. After a Weibo event is all input into the network, the output sequence *y*_*i*_={*y*_1_, *y*_2_,…, *y*_*N*_} is obtained.

Considering the time dependence of LSTM, an attention mechanism is introduced into the model. Taking the output of the hidden layer as the input of the attention layer, the formula of the attention layer is as follows:

(2) $$\begin{array}{c} e_{i}=\tanh\left(W_{w}y_{i}+b_{w}\right), \end{array}$$

where *W*_*w*_ and *b*_*w*_ represent the weight matrix and bias, respectively.

The output vector *y*_*i*_ of the attention mechanism is passed through a single-layer perceptron to obtain the intermediate vector *e*_*i*_ of the hidden layer state, and then, the paragraph level vector *v*_*w*_ is introduced to determine the weight *α*_*i*_ of the output vector *y*_*i*_ by calculating the similar values of the intermediate vectors *e*_*i*_ and *v*_*w*_ of the hidden layer state. The weight *α*_*i*_ is implemented by a softmax function:

(3) $$\begin{array}{c} \alpha_{i}=\frac{\exp\left(e_{i}^{T}v_{w}\right)}{\sum_{t}\exp\left(e_{i}^{T}v_{w}\right)}. \end{array}$$

The output sequence is given different weights, and the semantic feature *m*_*E*_ of the last event realized by weighted summation is as follows:

(4) $$\begin{array}{c} m_{E}=\sum_{t}\alpha_{t}y_{t}. \end{array}$$

When extracting statistical features, in order to obtain the same amount of information as semantic features, the statistical features are mapped into feature vectors with the same dimension as the output *m*_*E*_ through the full connection layer. The formula is as follows:

(5) $$\begin{array}{c} s=f\left(W_{s}\cdot f_{s}+b_{s}\right), \end{array}$$

(6) $$\begin{array}{c} f_{s}=f_{u}⊕f_{p}⊕f_{c}, \end{array}$$

where ⊕ indicates series operation, *f*_*u*_, *f*_*p*_, and *f*_*c*_, respectively, represent social features based on user information, social features based on communication content, and social features based on Weibo content.

Finally, the mapped statistical feature vector *s* and semantic feature vector are connected in series, and the two classification results are made through the Softmax layer. The prediction results are as follows:

(7) $$\begin{array}{c} p_{d}=\text{Softmax}\left\{m_{E}⊕s\right\}. \end{array}$$

The cross-entropy loss function is adopted in this model:

(8) $$\begin{array}{c} L=\sum_{d\in D}\left[y_{d}\log\;p_{d}+\left(1-y_{d}\right)\log\left(1-p_{d}\right)\right], \end{array}$$

where *d* is the sample, *D* represents the sample dataset, *y*_*h*_ represents the true value of the sample, and *p*_*d*_ is the predicted value of the sample. In the two classification results, 0 represents nonrumor and 1 represents rumor.

## 5. Experiment and Analysis

### 5.1. Simulation Environment Setting and Evaluation Index

The experiment environment adopts Linux system, and the environment configuration is shown in Table 1.

This study uses accuracy, precision, recall, and F1 score to evaluate the performance of the algorithm. The accuracy indicates the number of correctly classified samples, but when the positive and negative classes of the dataset are unbalanced, this index cannot accurately reflect the performance of the model, so it needs to be judged together with other indexes. Recall and precision will affect each other. Usually, one is high and the other is relatively low. In order to deal with this situation, the harmonic parameter F1 score of recall and precision is introduced. The calculation method of these four indicators is shown in formulas (9) to (12):

(9) $$\begin{array}{c} \text{Accuracy}=\frac{TP+TN}{TP+TN+FP+FN}, \end{array}$$

(10) $$\begin{array}{c} \text{Precision}=\frac{TP}{TP+FP}, \end{array}$$

(11) $$\begin{array}{c} \text{Recall}=\frac{TP}{TP+FN}, \end{array}$$

(12) $$\begin{array}{c} F1=\frac{2\times \text{Precision}\times \text{Recall}}{\text{Precision}+\text{Recall}}. \end{array}$$

For the rumor detection task, TP indicates that the tag is rumor and the classification result is rumor, TN indicates that the tag is nonrumor and the classification result is nonrumor, FP indicates that the tag is nonrumor, but the classification result is rumor, and FN indicates that the tag is rumor, but the classification result is nonrumor.

### 5.2. Comparison of Bid Evaluation Index Results of Each Model

In order to verify the effectiveness of the model, the proposed method is compared with the methods in [28, 29]. The original Weibo content and their comments were used for training, and the dataset was divided according to the ratio of 9 : 1 as training data and test data, respectively. The variation of accuracy, precision, recall, and F1 value with word2vec word vector is shown in Figure 6–9.

It can be seen from Figure 6–9 that the proposed model has greatly improved the accuracy, precision, recall, and F1 value compared with the methods in [28, 29]. When the word vector dimension is 300, the accuracy of the proposed method is 0.962, which is 4.113% and 1.477% higher than 0.924 in [28] and 0.948 in [29], respectively. The precision of the proposed method is 0.971, which is 5.773% and 1.996% higher than 0.918 in [28] and 0.952 in [29], respectively. The recall rate of the proposed method is 0.957, which is increased by 4.135% and 1.592% respectively compared with 0.919 in [28] and 0.942 in [29]. The F1 value of the proposed method is 0.964, which is increased by 5.011% and 1.795%, respectively, compared with 0.918 in [28] and 0.947 in [29]. The proposed method has advantages in the four indicators; this is because the proposed method integrates statistical features and semantic features. As a global feature in rumor detection, statistical features distinguish rumor and nonrumor attributes from the overall situation. However, the statistical feature is only the statistics of attributes, and the text semantics cannot be obtained. The text content can only be determined by special symbols or formats. Therefore, the combination of statistical features and semantic features expands the feature space in rumor detection and describes the distribution of data in the feature space to a greater extent, so as to improve the classification performance of the network. While literature [28] method and literature [29] method do not extract text features at a deep level. Based on the four experimental results, it can be seen that the proposed method has reached an advanced level in rumor detection, which shows the effectiveness of the model.

## 6. Conclusion

Aiming at the lack of feature extraction ability of rumor detection methods based on the deep learning model, this study proposes a rumor detection method based on deep learning in social network big data environment. The distributed word vector is used to encode text words, which improves the operation efficiency of the system in the case of a large number of corpus. In the optimization training stage, hierarchical softmax and negative sampling are used to improve the training efficiency. The multi-BiLSTM network and statistical feature fusion are constructed as the network structure of feature extraction to deeply extract text features and improve the classification efficiency. The attention mechanism is introduced to adjust the weight of the vector, which improves the efficiency and accuracy of task processing.

A problem in the existing research is that most of the existing datasets are for special events in a certain period of time, and the construction of data sets also depends on manual crawling and labeling. The dataset used in the experiment cannot be compared with the amount of information on the huge social network. In the follow-up work, we can try to use transfer learning to improve the generalization ability of the model.

## Figures and Tables

**Figure 1:** Flowchart of rumor detection based on deep learning.

**Figure 2:** Authorization process of OAuth agreement.

**Figure 3:** CBOW model.

**Figure 4:** Skip-gram model.

**Figure 5:** Multi-BiLSTM and statistical characteristics fusion model.

**Figure 6:** Comparison of accuracy of each model under Word2vec word vector.

**Figure 7:** Comparison of precision of each model under Word2vec word vector.

**Figure 8:** Comparison of recall of each model under Word2vec word vector.

**Figure 9:** Comparison of F1 value of each model under Word2vec word vector.

**Table 1:** Experimental environment configuration.

Items	Description
OS	Linux ubuntu 16.04
GPU	NVIDIA GeForce GTX 1080Ti
RAM	32G 1867MHZ DDR3

## Data Availability

The data used to support the findings of this study are included within the article.
